The article "Abdominal Cocoon: A Rare Complication of Peritoneal Dialysis in Chronic Kidney Disease" was retracted in 2024. Reasons: false authorship; unreliable results or conclusions; no approval from an author; concerns about the authorship.

# Abdominal Cocoon: A Rare Complication of Peritoneal Dialysis in Chronic Kidney Disease

**DOI:** 10.7759/cureus.20341

**Published:** 2021-12-11

**Authors:** Fatema Y Mohamed, Yasser H Alharbi, Mohammad N Almutairi, Nawaf A Azi, Alwaleed A Aljreas, Eman J Alkhaldi, Sulaiman H Alanazi, Abdullah T Alanazi, Mohammad S Alzahrany, Ahmed A Alali, Lujain H Alharthi, Rabab K Alkhalifah, Razan M Almarhoun, Hajar M Alkhadhabah, Faisal Al-Hawaj

**Affiliations:** 1 College of Medicine, Jordan University of Science and Technology, Irbid, JOR; 2 College of Medicine, Umm Al-Qura University, Mecca, SAU; 3 College of Medicine, Shaqra University, Shaqra, SAU; 4 College of Medicine, Royal College of Surgeons in Ireland, Dublin, IRL; 5 College of Medicine, King Saud bin Abdulaziz University for Health Sciences, Riyadh, SAU; 6 College of Medicine, Northern Border University, Arar, SAU; 7 College of Medicine, Medical University of Lublin, Lublin, POL; 8 College of Medicine, King Faisal University, Al-Ahsa, SAU; 9 College of Medicine, King Abdulaziz University, Jeddah, SAU; 10 College of Medicine, Imam Abdulrahman Bin Faisal University, Dammam, SAU

**Keywords:** case report, peritoneal dialysis, end-stage renal disease, abdominal pain, abdominal cocoon

## Abstract

The abdominal cocoon is a rare clinical entity characterized by a thick fibrocollagenous membrane encasing the intestinal loops. Despite its rarity, the abdominal cocoon is one of the most serious complications of peritoneal dialysis. We report the case of a 45-year-old man, with end-stage renal disease on peritoneal dialysis resulting from systemic lupus erythematosus, who presented to the emergency department with progressive abdominal pain for the last two weeks. The pain was associated with nausea, vomiting, abdominal distension, and decreased bowel motion. Upon examination, the vital signs were within the normal limits. Abdominal examination revealed a distended abdomen with generalized tenderness. There was evidence of ascites as indicated by the positive shifting dullness test. The bowel sounds were of increased frequency and intensity. The laboratory findings were non-contributory. The patient underwent an abdominal computed tomography scan that demonstrated a cluster of small intestinal loops in the middle of the abdomen with a surrounding thick and calcified membrane. This made the diagnosis of the abdominal cocoon. The patient underwent an operation to resect the fibrocollagenous membrane. The patient reported improvement after the operation. No recurrence was noted after three months of follow-up. Abdominal cocoon is a very rare complication of peritoneal dialysis. The diagnosis of abdominal cocoon should be kept in mind when the physician encounters a patient with peritoneal dialysis who presented with non-specific and unexplained gastrointestinal symptoms.

The article "Abdominal Cocoon: A Rare Complication of Peritoneal Dialysis in Chronic Kidney Disease" was retracted in 2024. Reasons: false authorship; unreliable results or conclusions; no approval from an author; concerns about the authorship.

## Introduction

Abdominal cocoon syndrome is a pathological condition that is characterized by the formation of a thick fibrocollagenous membrane encasing the intestinal loops [1]. It is a rare complication of continuous ambulatory peritoneal dialysis with a reported incidence of less than one per 1000 patient-years [2]. Despite its rarity, the abdominal cocoon is considered one of the most serious complications of peritoneal dialysis. The abdominal cocoon may result in intestinal obstruction and dialysis failure. Previous studies indicated high morbidity and mortality in patients with abdominal cocoons. The most important risk factors for the development of abdominal cocoon syndrome are the previous history of peritonitis and the duration of peritoneal dialysis [1]. Here, we present the case of a middle-aged man with an abdominal cocoon that developed after 15 years of peritoneal dialysis.

## Case presentation

We present the case of a 45-year-old man who presented to the emergency department complaining of vague abdominal pain for the last two weeks. The pain was generalized and colicky in nature. It was non-radiating. He reported that the pain was aggravated by any food intake. The pain was not related to posture. He attempted over-the-counter analgesics and antispasmodics, but he did not have any notable improvement. He scored the pain as 8 on the 10-point severity scale. The pain was disturbing his sleep pattern. It was associated with nausea, vomiting, abdominal distension, and bloating. He noted decreased bowel motion for the last one week. He reported that this is the first time for him to experience this pain.

The patient was diagnosed as having systemic lupus erythematosus at the age of 21 years. He developed lupus nephritis resulting in end-stage renal disease. He had peritoneal dialysis for the last 15 years. Further, the patient was known to have hypertension, dyslipidemia, and diabetes mellitus. These conditions were well-controlled with amlodipine 5 mg, metformin 1000 mg, atorvastatin 20 mg, and aspirin 75 mg. He did not undergo any previous surgeries. He was not known to have any allergies. He never smoked or consumed alcohol. The family history was remarkable for autoimmune diseases.

Upon examination, the patient appeared tired. His vital signs were within the normal range with a pulse rate of 88 bpm, respiratory rate of 16 bpm, temperature of 37.5°C, and blood pressure of 115/80 mmHg. The oxygen saturation was maintained. Abdominal examination revealed a distended abdomen with generalized tenderness. There was a shifting dullness indicative of ascites. No palpable masses were noted. Abdominal auscultation revealed bowel sounds of increased frequency and intensity. No hepatosplenomegaly. Examination of other systems was non-contributory.

The article "Abdominal Cocoon: A Rare Complication of Peritoneal Dialysis in Chronic Kidney Disease" was retracted in 2024. Reasons: false authorship; unreliable results or conclusions; no approval from an author; concerns about the authorship.

Initial laboratory examination revealed hemoglobin of 9.2 g/dL, leukocytes count of 8000/µL, and platelets count of 375,000/µL. The renal function tests revealed a creatinine level of 2.5 mg/dL and blood urea nitrogen of 51 mg/dL. The liver enzymes were within the normal range. The inflammatory markers, including erythrocyte sedimentation rate and C-reactive protein, were not elevated (Table 1).

**Table 1:** Summary of the results of laboratory findings

Laboratory Investigation	Unit	Result	Reference Range
Hemoglobin	g/dL	9.2	13.0–18.0
White Blood Cell	1000/mL	8.0	4.0–11.0
Platelet	1000/mL	375	140–450
Erythrocyte Sedimentation Rate	mm/hr.	14	0–20
C-Reactive Protein	mg/dL	8.2	0.3–10.0
Total Bilirubin	mg/dL	1.1	0.2–1.2
Albumin	g/dL	3.5	3.4–5.0
Alkaline Phosphatase	U/L	50	46–116
Gamma-glutamyltransferase	U/L	17	15–85
Alanine Transferase	U/L	16	14–63
Aspartate Transferase	U/L	18	15–37
Blood Urea Nitrogen	mg/dL	81	7–18
Creatinine	mg/dL	3.5	0.7–1.3
Sodium	mEq/L	138	136–145
Potassium	mEq/L	5.0	3.5–5.1
Chloride	mEq/L	105	98–107

Considering the aforementioned clinical signs and symptoms, the initial proposed diagnosis was an intestinal obstruction. The patient was resuscitated and parental analgesics were administered for pain control. Abdominal computed tomography was performed with intravenous contrast to confirm the diagnosis of intestinal obstruction and identify the etiology. The scan demonstrated a small intestinal loop in the center of the abdomen and surrounded by a thick calcified membrane. Further, the localized fluid collection was noted. Such findings conferred the diagnosis of an abdominal cocoon (Figure 1).

**Figure 1:** Selected axial CT image demonstrates a clustered small intestinal loop with the surrounding thick and calcified membrane (arrows). A localized fluid collection (asterisk) is also noted. CT: Computed tomography

Subsequently, the patient was prepared for emergency laparotomy. The operation was made under general anesthesia and the patient was placed in the supine position. During diagnostic exploration, the intestinal loops were found covered with a thick fibrocollagenous membrane. Meticulous dissection of the membrane was carried out. Complete excision of the membrane was performed. No bowel injury occurred during the dissection. The incisions were closed. The patient had an uneventful recovery. Histopathological examination of the excised membrane showed fibrocollagenous tissue (Figure 2). The loculated fluid was sent for culture and revealed no growth. Specifically, the fluid was negative for acid-fast bacilli. Following the operation, oral feeding was initiated gradually. The patient reported significant improvement in his symptoms. He was discharged after nine days of hospitalization. Peritoneal dialysis was discontinued after that and the patient started hemodialysis. After three months of follow-up, the patient remained asymptomatic with no evidence of recurrence.

The article "Abdominal Cocoon: A Rare Complication of Peritoneal Dialysis in Chronic Kidney Disease" was retracted in 2024. Reasons: false authorship; unreliable results or conclusions; no approval from an author; concerns about the authorship.

**Figure 2:** Histopathological examination of the excised membrane reveals fibrocollagenous tissue.

## Discussion

We reported the case of a middle-aged man with end-stage renal disease who developed abdominal cocoon syndrome after 15 years of peritoneal dialysis. The exact cause of abdominal cocoon is not fully understood. However, several hypotheses have been suggested about the possible pathogenesis [3]. The most accepted explanation is related to the peritoneal irritation and inflammation that results from the longstanding dialysis leading to the proliferation of the peritoneal lining cells [2]. Another alternative explanation is related to the upregulation of the renin-angiotensin system that results in the excessive formation of fibrin [3]. This fibrin deposition results in the formation of the thick membrane and abdominal cocoon. This hypothesis is supported by the finding that patients with angiotensin-converting enzyme inhibitors had a lower rate of fibrosis in the peritoneal lining [4].

Several risk factors have been reported to be associated with increased risk of abdominal cocoon in patients with peritoneal dialysis. It seems that the duration of peritoneal dialysis is the most significant factor [3]. In the present case, the duration was near 15 years after the onset of peritoneal dialysis. A multicenter study from Japan showed that the risk of abdominal cocoon was proportional to the total duration of peritoneal dialysis [5]. For example, the incidence of abdominal cocoon in patients with less than two years of peritoneal dialysis was <1% [5]. In addition, having episodes of severe bacterial or fungal peritonitis increases the risk significantly [2]. Further, the dialysate fluids may play a role as some components were found to increase the risk of peritoneal fibrosis [1].

Regarding the clinical presentation of the abdominal cocoon, it is frequently an asymptomatic disorder that develops after years of peritoneal dialysis [2]. The presenting symptoms are non-specific [5]. They include nausea, vomiting, and colicky abdominal pain. However, in the late stages of the abdominal cocoon, the patient may present with signs of intestinal obstruction, as in our case. No laboratory finding is associated with abdominal cocoon syndrome [3]. A computed tomography scan shows bowel tethering with peritoneal calcification [4]. However, normal imaging studies do not exclude the diagnosis. The management of abdominal cocoons includes medical and surgical options [2]. Tamoxifen and stopping the peritoneal dialysis can be attempted to improve the outcome in patients with abdominal cocoons [5]. However, since our patient had an acute presentation, surgical intervention was made.

The article "Abdominal Cocoon: A Rare Complication of Peritoneal Dialysis in Chronic Kidney Disease" was retracted in 2024. Reasons: false authorship; unreliable results or conclusions; no approval from an author; concerns about the authorship.

## Conclusions

Abdominal cocoon is a very rare complication of peritoneal dialysis. The diagnosis of abdominal cocoon should be kept in mind when the physician encounters a patient with peritoneal dialysis who presented with non-specific and unexplained gastrointestinal symptoms. A computed tomography scan is the key imaging modality to establish the diagnosis. However, laparotomy or laparoscopy is a confirmatory diagnostic procedure.
